The article "Patient satisfaction following treatment with micro‐focused ultrasound with visualization: A retrospective cross‐sectional study" was published in 2024. Journal: Skin Res Technol.

# Patient satisfaction following treatment with micro‐focused ultrasound with visualization: A retrospective cross‐sectional study

**DOI:** 10.1111/srt.13917

**Published:** 2024-08-09

**Authors:** Abrar Bukhari, Asem Shadid, Abdullah Al‐Omair, Ashjan Alheggi, Eman Abdulaziz Almukhadeb, Salma Y. Albarqawi

**Affiliations:** ^1^ Department of Dermatology College of Medicine Imam Muhammad Ibn Saud Islamic University (IMSIU) Riyadh Saudi Arabia; ^2^ Department of Dermatology King Fahad Medical City Riyadh Saudi Arabia; ^3^ Department of Dermatology Prince Sultan Military Medical City Riyadh Saudi Arabia; ^4^ Dermatology Department College of Medicine King Saud University Riyadh Saudi Arabia

**Keywords:** face and neck laxity, micro‐focused ultrasound, micro‐focused ultrasound with visualization (mfu‐v), ultherapy

## Abstract

**Background:**

There has been increased public interest in noninvasive skin tightening procedures that produce the best possible cosmetic outcomes. Micro‐focused ultrasound with visualization (MFU‐V) is a secure, efficient method of treating skin laxity approved by the FDA. Few studies have assessed patient satisfaction following MFU‐V.

**Materials and Methods:**

A retrospective cross‐sectional study was conducted between January 2022 and 2023. After obtaining the author's permission, a previously examined and published questionnaire was used to contact all participants (*n* = 98) who had received MFU‐V therapy in a private clinic in Riyadh, Saudi Arabia, between 2016 and 2020 via phone interview.

**Results:**

All 98 patients undergoing MFU‐V were female. About two‐thirds indicated they were satisfied or very satisfied with the results. Those receiving treatment around the eye and submentum reported lower satisfaction levels than those receiving therapy in other regions. The number of treatment locations and satisfaction were positively correlated. Patients treated by consultants rather than laser experts reported much higher satisfaction levels. Satisfaction and the amount of time for improvement to occur following treatment were correlated statistically. Pain and tingling were the most frequent adverse effects the respondents reported, followed by skin redness and swelling; however, adverse effects were not connected with satisfaction. Cost (78.6%) was cited as the main deterrent to seeking treatment again.

**Conclusion:**

MFU‐V, an FDA‐approved procedure, has proven effective and safe for treating facial and neck skin laxity. When patients are carefully selected and physicians properly trained, higher satisfaction is achieved.

## 1 INTRODUCTION

Skin photoaging has become common due to an increase in average life expectancy. It is clinically characterized by reduced cutaneous elasticity, roughness, and skin atrophy, appearances that can negatively affect an individual's quality of life.^1^ Public demand for noninvasive skin tightening techniques to achieve optimal cosmetic results, rapid recovery, and minimal risk has increased. Recently, multiple new devices have been proposed to treat skin laxity.^2^

The article "Patient satisfaction following treatment with micro‐focused ultrasound with visualization: A retrospective cross‐sectional study" was published in 2024. Journal: Skin Res Technol.

While both HIFU (High‐Intensity Focused Ultrasound) and MFU‐V; Ultherapy (Micro‐focused ultrasound with visualization) utilize ultrasound technology to stimulate collagen production, they serve distinct purposes. HIFU is a broader term encompassing various medical applications, including non‐invasive cancer treatment and uterine fibroid management, where high‐intensity ultrasound energy is concentrated to destroy abnormal cells. In contrast, Ultherapy is a specific aesthetic application of HIFU that delivers micro‐focused ultrasound energy to precise skin layers, triggering collagen production for skin tightening and lifting. Unlike HIFU, Ultherapy employs ultrasound imaging to visualize and target specific tissue depths, ensuring precise treatment delivery.^3^, ^4^, ^5^ Micro‐focused ultrasound with visualization (MFU‐V; Ultherapy) received FDA approval in 2009 and emerged as a safe, effective means of treating skin laxity. The difference between MFU‐V and other preexisting skin tightening technologies is its ability to engage deeper tissues while sparing the above epidermis.^5^

Micro‐focused ultrasound (MFUS) delivers focused heating up to 60°C, producing a small thermal coagulation zone (less than 1 mm) to heat tissue at specific depths that reach from the mid‐to‐deep dermis into the superficial musculoaponeurotic system, subsequently leading to collagen denaturation, contraction, and new collagen formation.^6^

Counseling regarding realistic expectations for MFUS is essential, as clinical studies have shown that it produces acceptable results, but it gradually subsides in 3–6 months.^7^ Based on recent reviews, few studies have assessed patient satisfaction following treatment with MFU‐V.^8^ The present study aimed to determine patient safety, efficacy, and satisfaction with their aesthetic results following MFUS treatment and the association between medical practitioners’ qualifications and the satisfaction rate. It attempted to identify why patients stated they would not undergo this procedure in the future.

## 2 MATERIALS AND METHODS

In a retrospective cross‐sectional study performed between January 2022 and January 2023, all patients (*n* = 98) who had undergone MFU‐V treatment in a private clinic in Riyadh, Saudi Arabia, between 2016 and 2020 were contacted via a phone interview. Participation was voluntary, and informed consent was obtained. The study followed the code of ethics of the Declaration of Helsinki. The institutional review board approval number (HAPO‐01‐R11) was obtained in advance by the Ethics and Research Committee of Al‐Imam Muhammad Ibn Saud Islamic University, College of Medicine. Informed consent was obtained from all participants.

The article "Patient satisfaction following treatment with micro‐focused ultrasound with visualization: A retrospective cross‐sectional study" was published in 2024. Journal: Skin Res Technol.

A previously published questionnaire was validated and used after obtaining author approval.^7^ Since the questionnaire was originally written in English, it was translated into Arabic. The first part of this electronic questionnaire included demographic characteristics, and the second part assessed the participants’ experience and outcome regarding MFUS, including the site of treatment, the number of regions, post‐treatment follow‐up appointments, the qualifications of the person who performed the treatment, satisfaction with the treatment results, side effects, and reasons for not considering the treatment again.

Statistical analysis was performed using R *v* 3.6.3. Counts and percentages were used to summarize categorical variables. The mean ± standard deviation and the median interquartile range were used to summarize the continuous standard and non‐normal variables, respectively. A chi‐square test of independence was used to assess the association between categorical variables. Hypothesis testing was performed at a 5% level of significance.

## 3 RESULTS

A total of 98 patients underwent MFU‐V, all of whom were female. Of these, 91 (92.9%) were aged 35−50, and 6 (6.12%) were aged 51−60. Most respondents had MFU‐V applied to the submentum area (93.9%), and more than three‐quarters (81.6%) had MFU‐V applied around the eyes. Less than one‐quarter received treatment on the chin (23.5%) and neck (19.4%) (Figure 1(A)). The results showed that 19 (19.4%) of the respondents received treatment in only one region, compared to 13 (13.3%) in all four regions. More than half of the respondents received treatment in two regions (Figure 1 (B)).

**FIGURE 1:** (A) Site of MFU‐V treatment, (B) number of regions that received MFU‐V.

Three‐quarters (76.5%) of the respondents did not have scheduled post‐treatment follow‐up appointments, while 19.4% had one, and 4.08% had two. Of the 23 respondents who had follow‐up appointments, more than three‐quarters (78.3%) attended one. The treatment was performed by a laser specialist in 17.3% of the respondents and by a consultant in the remaining 82.7% (Table 1). Approximately half of the respondents stated that friends (55.1%) and family (51%) had noticed the post‐treatment results. Approximately one‐third of the respondents (30.6%) noted that no one had noticed the post‐treatment results (Figure 2).

The article "Patient satisfaction following treatment with micro‐focused ultrasound with visualization: A retrospective cross‐sectional study" was published in 2024. Journal: Skin Res Technol.

**TABLE 1:** Participants’ experience with MFU‐V.

	*N *= 98
**Post‐treatment follow‐up appointments scheduled**:	
None	75 (76.5%)
1	19 (19.4%)
2+	4 (4.08%)
**Post‐treatment follow‐up appointments attended**	
1	18 (78.3%)
2	1 (4.35%)
I attended all the appointments	1 (4.35%)
I did not attend an appointment	3 (13.0%)
**The last post‐treatment follow‐up appointment attended**	
1 Week	2 (8.70%)
1 Month	3 (13.0%)
3 Months	4 (17.4%)
More than 3 months	14 (60.9%)
**Qualifications of the person who performed the treatment**	
Consultant	81 (82.7%)
Laser specialist	17 (17.3%)
Data were summarized using counts and percentages	

**FIGURE 2:** Responses to “Who noticed the post‐treatment results?”.

Approximately two‐thirds of the respondents were either satisfied or very satisfied with the treatment outcomes, while about one‐quarter (21.4%) were neutral. The expectations regarding treatment outcomes were met in 43.9% of the patients, and the expectations were exceeded in approximately 25% of patients. About one‐third (35.7%) of the respondents began noticing a difference 1 month after the session, and approximately one‐quarter began noticing a difference 3 or more months afterward (24.5%). Only 57.1% of the respondents considered undergoing treatment again (57.1%), and three‐quarters (71.4%) mentioned that they would recommend the treatment for someone else (Table 2). The most common side effects experienced by the respondents were pain and tingling (57.9%), followed by skin redness (47.4%) and swelling (26.3%) (Figure 3 (A)). The most common reason for not considering treatment again was cost (78.6%), followed by the results not meeting expectations (59.5%). Other reasons included results not lasting as long as expected (38.1%) and side effects (2.4%) (Figure 3 (B)).

**TABLE 2:** Outcomes of MFU‐V.

	*N = 98*
**Satisfaction toward the treatment results**:	
Very dissatisfied	5 (5.10%)
Dissatisfied	9 (9.18%)
Neutral	21 (21.4%)
Satisfied	40 (40.8%)
Very satisfied	23 (23.5%)
**Results matched the expectations**	
The results were much poorer than I expected	8 (8.16%)
The results were poorer than I expected	22 (22.4%)
Met expectations	43 (43.9%)
Exceeded expectations	22 (22.4%)
Far exceeded expectations	3 (3.06%)
**Time to start noticing the difference**	
During the session	18 (18.4%)
After 1 week	21 (21.4%)
After 1 month	35 (35.7%)
After 3 months	10 (10.2%)
More than 3 months	14 (14.3%)
**Consider undergoing the treatment again**	
No	42 (42.9%)
Yes	56 (57.1%)
**Recommend the treatment for someone else**	
No	28 (28.6%)
Yes	70 (71.4%)
Data were summarized using counts and percentages	

**FIGURE 3:** (A) Side effects experienced by respondents, (b) reasons for not considering the treatment again.

The article "Patient satisfaction following treatment with micro‐focused ultrasound with visualization: A retrospective cross‐sectional study" was published in 2024. Journal: Skin Res Technol.

The results showed that a longer time before noticing improvement following treatment was associated with lower satisfaction with treatment (*r* = −0.456, *p* < 0.001), less likelihood of recommending treatment to someone else (*r* = −0.499, *p* < 0.001), and less likelihood of the results meeting expectations (*r* = −0.515, *p* < 0.001) (Figure 4). However, age and the time of the last follow‐up appointment were not significantly associated with satisfaction. Satisfaction was significantly higher among the respondents who had received treatment around the eyes than in any other area (*p* = 0.006). Similarly, the respondents who had received treatment in the submentum indicated more satisfaction than the respondents who had received treatment in other areas (*p* = 0.004).

**FIGURE 4:** Correlations between satisfaction with MFU‐V.

Satisfaction was significantly higher among respondents who had received treatment by a consultant than by a laser specialist (71.6% vs. 29.4% were satisfied, respectively, *p* = 0.002). A statistically significant linear trend was observed in the association between the time it took to notice a difference after treatment and satisfaction, with 94% of respondents who had experienced improvement during the session reporting satisfaction, compared to only 7.14% who had observed improvement after more than 3 months following the session (Table 3). However, experiencing side effects after the session was not associated with satisfaction. The respondents who reported that the post‐treatment results were noticed by family and friends (88%) indicated higher satisfaction than the respondents whose post‐treatment results were not noticed (13.3%). The duration of the treatment effects was significantly associated with satisfaction (*p* = 0.002), with 87.1% satisfaction reported by respondents whose treatment effects lasted 12 months. This rate was much higher than the 53.8% satisfaction rate among patients whose treatment effects lasted 6 months (Figure 5(A)). A positive association was found between the number of regions that received treatment and satisfaction (*p* = 0.01) (Figure 5(B)).

**TABLE 3:** Factors associated with satisfaction with MUF‐V results.

	Dissatisfied	Neutral	Satisfied	*p*
	***N = 14***	***N = 21***	***N = 63***	
**Age**:				0.109
35−50 years	11 (12.1%)	20 (22.0%)	60 (65.9%)	
51−60 years	3 (50.0%)	1 (16.7%)	2 (33.3%)	
61 years and older	0 (0.00%)	0 (0.00%)	1 (100%)	
**Treatment areas**	–	–	–	–
Around the eyes	12 (15.0%)	12 (15.0%)	56 (70.0%)	0.006
Submentum	10 (10.9%)	20 (21.7%)	62 (67.4%)	0.004
Chin	3 (13.0%)	2 (8.70%)	18 (78.3%)	0.220
Neck	1 (5.26%)	2 (10.5%)	16 (84.2%)	0.183
**Was the last post‐treatment follow‐up appointment attended?**				0.597
1 Month	0 (0.00%)	0 (0.00%)	3 (100%)	
1 Week	0 (0.00%)	0 (0.00%)	2 (100%)	
3 Months	2 (50.0%)	0 (0.00%)	2 (50.0%)	
More than 3 months	2 (14.3%)	1 (7.14%)	11 (78.6%)	
**Started noticing the difference**				<0.001^a^
During the session	0 (0.00%)	1 (5.56%)	17 (94.4%)	
After 1 week	0 (0.00%)	4 (19.0%)	17 (81.0%)	
After 1 month	1 (2.86%)	10 (28.6%)	24 (68.6%)	
After 3 months	3 (30.0%)	3 (30.0%)	4 (40.0%)	
After more than 3 months	10 (71.4%)	3 (21.4%)	1 (7.14%)	
**Experienced side effects after the treatment session**				0.647
No	10 (12.7%)	17 (21.5%)	52 (65.8%)	
Yes	4 (21.1%)	4 (21.1%)	11 (57.9%)	
**How long did the treatments results last?**				0.002
12 Months	0 (0.00%)	4 (12.9%)	27 (87.1%)	
18 Months	1 (50.0%)	0 (0.00%)	1 (50.0%)	
6 Months	13 (20.0%)	17 (26.2%)	35 (53.8%)	
**Would you consider undergoing the treatment again?**	0 (0.00%)	0 (0.00%)	1 (100%)	<0.001
No	14 (33.3%)	16 (38.1%)	12 (28.6%)	
Yes	0 (0.00%)	5 (8.93%)	51 (91.1%)	

^a^ Data were summarized using counts and percentages. Analysis was performed using the chi‐square test of independence.

The article "Patient satisfaction following treatment with micro‐focused ultrasound with visualization: A retrospective cross‐sectional study" was published in 2024. Journal: Skin Res Technol.

**FIGURE 5:** (A) Relationship between the time before noticing a difference and satisfaction, (B) association between the number of regions that received treatment and satisfaction.

## 4 DISCUSSION

The therapeutic use of ultrasound in the aesthetic field focuses on a particular area of the body to penetrate deeper into a tissue, encourages thermal coagulation, and improves skin remolding, avoiding the unfavorable post‐procedural consequences seen with other techniques, such as carbon‐dioxide laser resurfacing.^9^ MFU‐V is a minimally invasive, safe, effective cosmetic therapy approved by the FDA. It is routinely used in dermatological clinics worldwide.^7^, ^8^

MFU‐V treats face and neck laxity effectively, particularly in the first 6 months of therapy. Some studies have used adjuvant therapy, such as calcium hydroxylapatite (CaHA). However, because CaHa is licensed for use as a monotherapy to address face and neck laxity, treatment outcomes may differ from those obtained with MFU‐V alone. Higher satisfaction ratings were achieved with a combined therapy using MFU‐V and diluted or hyper‐diluted CaHA. Around half of the patients were described as “much improved” or “very much improved” on days 30 and 90.^8^ In the present study, 35.7% of participants reported noticing a difference 1 month after the session, while 24.5% reported noticing it after 3 months or more. The results also showed that lower treatment satisfaction, a lower likelihood of recommending treatment to a friend, and a lower likelihood of results meeting expectations were associated with a longer time to notice a difference post‐treatment. The correlation between the time it took to notice a difference after treatment and satisfaction was statistically significant, with 94% of respondents indicating satisfaction when they saw improvement during the session compared to only 7.14% when they saw improvement after more than 3 months.

The article "Patient satisfaction following treatment with micro‐focused ultrasound with visualization: A retrospective cross‐sectional study" was published in 2024. Journal: Skin Res Technol.

In previous studies, satisfaction evaluation was often a source of concern because the subjective evaluations of MFU‐V devices have various drawbacks. First, the subjective scoring approach provides a non‐anonymous platform with the potential to skew the results due to patient interpretation differences. Furthermore, there is currently no anonymous validating subjective grading method for the treatment of face and neck laxity. However, data on subjective scoring systems, including the Patient Satisfaction Questionnaire, Subjective Global Aesthetic Improvement Scale, the three‐point scoring system, and self‐developed scoring, have been well established and validated for patients with face and neck laxity who have undergone MFU‐V. However, all of these scoring systems use non‐anonymous data that may influence patients’ responses and lead to doctor bias.^6^, ^10^

The most adverse effects found in earlier research were moderate bruising, redness, and pain. None of the subjects recorded any major adverse effects. In one case, a burn occurred because of improper application of the probe.^8^ In our sample, adverse effects following the session did not correlate with satisfaction. Additionally, there was a strong correlation between patient satisfaction and the credentials of the treating physician, with dermatologist‐treated patients reporting more significant levels of satisfaction than laser specialist‐treated patients (71.6% vs. 29.4%).

This study's main strength is that it can provide physicians with an understanding of patient satisfaction and how higher medical credentials may affect it. Yet this study has limitations. Since no male subjects underwent this procedure in the facility in which the study was undertaken, the sample comprised 100% female subjects. Moreover, the study was conducted using only Arabic participants, thus excluding other races.

## 5 CONCLUSION

MFUS with visualization is an FDA‐approved system that has proven effective and safe for treating skin laxity on the face and neck. Respondents who received treatment around the eyes and submentum reported higher satisfaction than those who received treatment in other locations. Satisfaction and the number of treated regions were positively correlated. A significant difference in satisfaction was found between respondents treated by consultants and those treated by laser specialists. The correlation between the time it took to notice n improvement after treatment and satisfaction was statistically significant. Pain and tingling were the most common side effects, followed by redness and swelling of the skin. It is recommended that patients be selected at the right time, under the guidance of a qualified physician, and are educated regarding the length of time and expectations for the results. In addition, a proper satisfaction evaluation must be implemented.

The article "Patient satisfaction following treatment with micro‐focused ultrasound with visualization: A retrospective cross‐sectional study" was published in 2024. Journal: Skin Res Technol.

## CONFLICT OF INTEREST STATEMENT

The authors declare no conflicts of interest.

## ETHICS STATEMENT

The declaration of Helsinki's code of ethics was adhered to in this investigation. Al‐imam Muhammad Ibn Saud Islamic University, College of Medicine's Institutional Review Board of Ethics and Research Committee approved the project under approval number hapo‐01‐r11.

## Data Availability

All data generated or analyzed during this study are included in this article. Further enquiries can be directed to the corresponding author.
